This article has been retracted.

# Cognitive Computation in Ideological and Political Classroom Teaching Based on Digital Sensor Technology

**DOI:** 10.1155/2022/8723327

**Published:** 2022-07-18

**Authors:** Hong Cai

**Affiliations:** College of Marxism, Inner Mongolia University of Finance and Economics, Hohhot, Inner Mongolia 010000, China

## Abstract

Numerous new ideas and concepts have changed the behavior and value orientation of university students as a result of the internet's rising popularity on college campuses. This study performs research on digital sensor technologies in order to enhance the intelligent effect of ideological and political classroom instruction. In addition, this study combines the fast Fourier transform principle to enhance digital sensor technology, digital sensor and cognitive computation technology to investigate the ideological and political classroom teaching process, and the actual situation of the ideological and political teaching to digitally process the ideological and political teaching process. In addition, this study employs sensor technology to convey data and digital sensor technology to increase the quality of ideological and political classroom instruction by enhancing the traditional teaching paradigm. In addition, on this premise, this study conducts a performance evaluation of the system, primarily focusing on the digital effect and the enhancement of ideological and political teaching quality. In conclusion, this study proves its teaching system through test research. According to the test results, the intelligent teaching method described in this study has a certain practical effect.

## 1. Introduction

The ideological and political theory courses of colleges and universities undertake the important task of ideological and moral education for college students, and help college students to establish a correct outlook on the world, life, values, ethics, and legal system under the guidance of scientific theories. Judging from the current situation investigation and analysis, the current overall response of college students to “ideological and political courses” is not ideal. The current ideological and political education in colleges and universities in my country is basically the implementation of a “unilateral policy,” that is, the main method is indoctrination and narration, which lacks interest, diversity, and abstraction. As a result of “indoctrination” with uninteresting and meaningless theories, some college students with higher education often have clear discrepancies in their ideological, political, and ethical standards, and beliefs. Furthermore, these kids' “main beliefs” are evident, yet their daily behaviors are aggravating. There are many reasons for the lack of vitality and vitality in the teaching of “ideological and political courses,” and the combination of many factors has formed the current situation of disconnection between the teaching and learning of “ideological and political courses.” Therefore, how to make students pay attention to ideological and political courses, get innovative thinking and innovative spirit training and training in ideological and political courses, and make our ideological and political education receive good results is a topic that every ideological and political teacher should think about [1].

With the rapid development of educational informatization, colleges and universities, as the forefront of teaching and research and the main front of student scientific research activities, are also making great strides to achieve the goal of informatization campus [2]. Among them, information-based teaching provides strong support for characteristic teaching in colleges and universities, and it is also the key to the overall construction of colleges and universities. It can be seen that the task of optimizing the campus network topology system structure and accelerating the pace of building an informationized campus is imminent [3]. The application of digital sensor technology has enriched the teaching tools of high school chemistry and integrated the experimental methods and experimental contents. The application of digital sensor technology has also promoted the change in teachers' teaching concepts [4]. In the three-dimensional teaching goals proposed in the modern education reform, students must not only learn knowledge and skills, but also through the learning process, learn scientific thinking and methods, and acquire emotional attitudes and values. Moreover, the introduction of digital sensor technology not only allows students to acquire knowledge, but also more importantly, through the process of chemical experiment inquiry, to learn scientific thinking and research methods, and to enhance students' practical ability. In addition, it better embodies the teaching philosophy of learning as the main body and teaching as the leading factor, and at the same time stimulates students' interest in chemistry learning, cultivates their pragmatic, rigorous, and scientific attitude, and enhances students' scientific literacy. So far, most schools have conducted research studies on digital sensor technology instruments, but they have not yet fully utilized the advantages of digital sensor technology. How to combine digital sensor technology with high school chemistry experiments and how to combine digital sensor technology with student experiments will be the focus of the next research. This study applies digital sensor technology to ideological and political classroom teaching, constructs a system functional structure, and verifies the effect of this teaching method.

This study uses sensor technology to convey data, and digital sensor technology, with the goal of improving the quality of ideological and political classroom learning by enhancing the paradigm of traditional teaching. In addition, on the basis of this premise, this study does a performance evaluation of the system, especially concentrating on the digital effect and the improvement of the quality of ideological and political instruction. In conclusion, this study demonstrates that its instructional methodology is supported by test research. The findings of the tests indicate that the intelligent teaching strategy that is discussed in this study does have some effect in the real world.

## 2. Related Work

As early as the 20th century, foreign developed countries began to focus on integrating many advanced technologies into the education of various subjects such as mathematics, physics, chemistry, and biology, and such as ICT (information and communication) and sensor technology. The integration of computer-centric information and communication technology and education has become an important trend in education reform, and it is also a powerful driving force for education reform in Western countries (including education goals, content, methods, and forms) [5].

Western schools have invested a lot of money in ICT research. Literature [6] studied why teachers participate in the training of information and communication technology projects, and found that in addition to their interest, it is more important to help their teaching. Lifelong learning is particularly important in the rapidly developing modern society. Therefore, ICT on-the-job training conforms to the requirements of the modern social and cultural environment.

Sensor technology is one of the three key technologies of acquisition, processing, and dissemination in information technology, and many countries classify it as a cutting-edge technology. The United States claims that the world has entered the sensor era, and Japan ranks sensor technology as the top ten technologies [7]. Since the 1980s, it has been widely used in various levels of education in foreign developed countries. Sensing technology is used in science teaching and experimental investigation in middle schools in the United States, Singapore, and some European countries and regions [8]. Since the development of sensor technology abroad, the application research in chemical experiments has become more and more mature, such as carbon dioxide sensor, dissolved oxygen sensor [9], and so on. Literature [10] pointed out that self-sustaining research on oxygen sensors has led to the development of various applications and different performance characteristics of the sensors. In order to meet the needs of teachers and students, the United States has published many books on the application of digital sensor technology to middle school chemistry experiments, such as chemistry with computer (31 experiments), advanced chemistry with vernier (35 experiments), science with handhelds (experiment-attached CD), and chemistry with calculators (36 experiments). These experimental books show that the development of digital sensor technology in the United States is relatively mature, and it has a positive guiding role in the development and use of digital sensor technology in our country [11].

A digital experiment based on digital sensor technology is one that employs a computer as a platform to carry out chemical tests in real time. It incorporates a wide range of modern scientific and technological breakthroughs, such as simulation trials, sensor experiments, and multimedia displays. Because it is still in its early stages of development, the present name of this technology in our country is not standardized. The names of the categories of technology are “sensing technology,” “handheld technology,” and “handheld technology.” The names of the secondary device categories are “digital exploration laboratory,” “digital information system (abbreviated as DIS),” “handheld laboratory” [12], and so on. Due to the intuitive “digital” feature of the technology and the important role played by its key component “sensor,” it is named digital sensor technology. Digital sensor technology was introduced to our country at the beginning of this century, and more and more front-line teachers began to study digital sensor technology. In order to objectively understand the hotspots and key points of the research on chemistry experiment teaching in middle schools in our country, the literature [13] used relevant software and tools to sort out and analyze the research results of a large number of existing middle school chemistry experiment teaching and drawled the hotspot knowledge map of its research.

Virtual reality technology has been out of the laboratory in the 1970s, has been used by people in the application market, and has been unanimously favored by everyone. Therefore, individual countries in the world that have conducted VR research, especially developed countries, have taken the lead in conducting extensive research and discussions on related projects. Some schools abroad have used VR equipment to do some remote teaching activities. Students have provided feedback indicating that the impact of learning can be more concentrated in some classes due to the immersion that occurs during the process of using VR equipment. On the other hand, the experience of teaching in a traditional classroom setting, such as taking notes, needs to be more technically correct. However, it is understandable that if it is truly mature and applied, VR will bring breakthrough progress for practical operation and experimental teaching [14].

## 3. The Principle and Analysis of Fast Fourier Transform

The angular frequency of the periodic signal *x*(*t*) is *ω* = 2*πf* = 2*π*/*T*; the period is *T*; and its FFT is transformed into [15] the following:

(1) $$\begin{array}{c} x\left(t\right)=A_{0}+A_{1}\cos\;\omega t+B_{1}\sin\;\omega t+A_{2}\cos\;2\;\omega t+B_{2}\sin\;2\;\omega t+\ldots \\ =A_{0}+\sum_{h=1}^{\infty }A_{h}\cosh\;\omega t+\sum_{h=1}^{\infty }B_{h}\sinh\;\omega t. \end{array}$$

In the above formula, *A*_0_=1/*T*∫_−*T*/2_^*T*/2^*f*(*t*)d*t* represents the DC quantity of the periodic signal, and the coefficients of the expression after the FFT transformation of the periodic signal are Ah and Bh.

(2) $$\begin{array}{c} Ah\;=\frac{2}{T}\int_{-T/2}^{T/2}f\left(t\right)\cosh\;\omega tdt,\;h=1,2,\ldots \\ Bh\;=\frac{2}{T}\int_{-T/2}^{T/2}f\left(t\right)\sinh\;\omega t\text{d}t,\;h=1,2,\ldots \end{array}$$

The above formula (1) can be simplified as follows:

(3) $$\begin{array}{c} x\left(t\right)=C_{0}+\sum_{h=1}^{\infty }C_{h}\cos\left(h\omega t+\varphi_{h}\right). \end{array}$$

In the time domain, two consecutive signals are multiplied, the result of the multiplication is Fourier transformed, which is equal to the Fourier transform of the respective sequence, and then, the convolution operation is performed. After the above analysis, the infinite signal *x*ʹ(*n*) is DTFT transformed into the following:

(4) $$\begin{array}{c} X\left(e^{jw}\right)=\text{DTFT}\left(x^{\prime }\right). \end{array}$$

In the above formula (3), *C*_0_=*A*_0_ represents the direct current, $C_{h}=\sqrt{A_{h}^{2}+B_{h}^{2}}$ represents the magnitude of the periodic signal in the *h*th harmonic amplitude, and *φ*_*h*_=arc tan(*A*_*h*_/*B*_*h*_) represents the magnitude of the periodic signal in the *h*^th^ harmonic phase. When we sample the signal, we can set *N* sampling points, and the sampling frequency is *f*_*s*_. By sampling the periodic signal, the expression of the signal in the time domain can be obtained, which is [16] the following:

(5) $$\begin{array}{c} x\left(n\right)=C_{0}+\sum_{h=1}^{\infty }C_{h}\cos\left(h\omega \frac{n}{f_{s}}+\varphi_{h}\right),\;n=0,1,\ldots ,N-1. \end{array}$$

When performing FFT transformation on a periodic signal, it is necessary to perform transformation analysis not only in the time domain but also in the frequency domain, so that the characteristics of the signal can be better understood. If a continuous signal *x*(*t*) satisfies the Dirichlet condition, then

(6) $$\begin{array}{c} \int_{-\infty }^{+\infty }\left|x\left(t\right)\right|\text{d}t<\infty . \end{array}$$

Then, the Fourier transform FFT of *x*(*t*) is as follows:

(7) $$\begin{array}{c} X\left(j\omega \right)=\int_{-\infty }^{+\infty }x\left(t\right)e^{-j\omega t}\text{d}t. \end{array}$$

Its inverse Fourier transform (IFFT) is as follows:

(8) $$\begin{array}{c} x\left(t\right)=\frac{1}{2\pi }\int_{-\infty }^{+\infty }X\left(j\omega \right)e^{j\omega t}\text{d}t. \end{array}$$

Equations (7) and (8) are a set of FFT transformation and inverse FFT transformation, where the FFT transformation obtains the signal's spectral function, and the inverse FFT transformation obtains the value of the signal at each time *t*. When we uniformly sample the signal, what we need is the value of each point of the signal. By performing a discrete Fourier transform on an infinitely long signal, we can get [17] the following:

(9) $$\begin{array}{c} X\left(j\omega \right)=\sum_{n=-\infty }^{+\infty }x\left(n\right)e^{-j\omega n}. \end{array}$$

The above formula expresses the result obtained by the DTFT transformation of an infinitely long signal. This is mainly suitable for theoretical analysis and not suitable for calculation and analysis on a computer. Therefore, we need a signal of finite length so that it can be applied in practice. We apply the above formula (9) to a transformation, the variable *ω* = 2*πk*/*N* is brought into it to obtain the following:

(10) $$\begin{array}{c} X\left(k\right)=\sum_{n=0}^{N-1}x\left(n\right)e^{-j\left(2\pi /N\right)},\;k=0,1,\ldots ,N-1. \end{array}$$

Formula (10) is the discrete Fourier transform DFT of a signal *x*(*n*) of finite length, and its inverse discrete Fourier transform is as follows:

(11) $$\begin{array}{c} x\left(n\right)=\frac{1}{N}\sum_{n=0}^{N-1}X\left(k\right)e^{j\left(2\pi /N\right)nk},\;n=0,1,\ldots ,N-1. \end{array}$$

The above equations (10) and (11) are the DFT and IDFT of the finite-length signal *x*(*n*), where the DFT transform obtains the discrete spectrum function of the signal. The FFT algorithm is widely used in signal analysis. This study applies the FFT algorithm to the time grid signal acquisition to reduce the error of its measurement.

When performing FFT transformation on a continuous signal, in actual operation, only a limited-length signal can be intercepted for analysis. In this process, some errors will be brought, that is, spectrum leakage and fence effect.

### 3.1. Spectrum Leakage

Since only a period of time can be selected for analysis in actual engineering applications, in essence, the signal is multiplied by a rectangular window function to obtain a finite-length signal *x*(*n*). That is, the infinite signal *x*ʹ(*n*) is limited to 0 ≤ *n* ≤ *N* − 1. The frequency density function of the rectangular window is [18] as follows:

(12) $$\begin{array}{c} W_{R}\left(e^{j\omega }\right)=\text{DTT}\left(R_{N}\left(n\right)\right)=\frac{\sin\left(\omega N/2\right)}{\sin\left(\omega /2\right)}e^{-j\left(N-1/2\right)\omega }. \end{array}$$

In the time domain, two consecutive signals are multiplied, and the result of the multiplication is Fourier transformed, which is equal to the Fourier transform of the respective sequence, and then, the convolution operation is performed. After the above analysis, the infinite signal *x*ʹ(*n*) is DTFT transformed into the following:

(13) $$\begin{array}{c} X\left(e^{j\omega }\right)=\text{DTFT}\left(x^{\prime }\left(n\right)R_{N}\left(n\right)\right)=\frac{1}{2\pi }\int_{-\pi }^{\pi }X^{\prime }\left(e^{-j\theta }\right)W_{R}\left(e^{j\left(\omega -\theta \right)}\right)\text{d}\theta . \end{array}$$

Figure 1 shows the schematic diagram of frequency leakage. In Figures 1(a) and 1(b), it can be seen that there is no leakage of the spectrum when an infinitely long signal is converted by DTFT. However, in Figures 1(c) and 1(d), it can be seen that after the infinite signal is truncated, when the obtained finite signal is subjected to DTFT conversion, the leakage of the spectrum occurs [19].

### 3.2. Fence Effect

When using the FFT algorithm to analyze a signal, the continuous frequency spectrum of the signal must be discretely sampled at equal intervals. When the continuous spectral density function *X*(*jω*) is uniformly sampled, *X*(*k*) is obtained through discrete Fourier transform (DFT).  Figure 2 shows the schematic diagram of the fence effect. In the process of signal sampling, ideally the sampled spectrum is just the desired target spectrum so that the parameter values of the spectrum can be easily obtained. However, in actual situations, it is very difficult for the sampled spectrum to coincide with the target spectrum. In fact, there will be a certain distance from the target curve. In this way, many frequency points will be lost and a fence effect will appear. As shown in Figure 2(a), in an ideal situation, the sampled spectral line *k*_*p*_ is just the desired target spectral line *K*_0_ so that the parameter values of the *K*_0_ spectral line can be easily obtained. As shown in Figure 2(b), in the actual situation, the sampled spectral line *k*_*p*_ and the desired target spectral line *K*_0_ are not together, and there is a certain distance. In order to reduce the fence phenomenon, we can appropriately increase the number of sampling points, which can reduce the distance between the sampled spectral lines, make the sampled spectral lines closer to the target spectral line, and improve the sampling accuracy [20].

## 4. Ideological and Political Classroom Teaching System Based on Digital Sensor Technology

The ideological and political education digital resource platform's technical route primarily consists of resource content selection, audience analysis, environment configuration, development tool configuration, framework construction, and the processing of digital resource material, graphic design, network addition of materials, testing and evaluation, modification, optimization, and other 13 technical links. Through the analysis of the technical route, the system construction resource platform is shown in Figure 3 [21].

A blueprint for the creation of a digital resource platform for the ideological and political education of students in the classroom is conceived and developed on the basis of unmistakable design principles and concepts. The resource library system and the support system for the platform are the primary components of the model. The primary components of the support system are the learning system and the teaching system, both of which encompass various aspects of education and scientific research and text resource library, picture resource library, video resource library, animation resource library, and resource retrieval system with the theme of each resource library that are the main components of the interactive system that make up the resource library system. Together, these components form a resource data platform that integrates storage, calling, and management. There is a connection between each resource library and network system, and between the learning system, teaching system, teaching resource editing system, and the production system. The back-end management of the system platform must meet stringent standards if the digital resource platform for ideological and political education in the classroom is to function without hiccups. Ideological and political classroom teaching digital resource platform management system includes teaching management (teacher management, student management, etc.), resource library management (text, pictures, video, animation, data and other resources, network teaching resource management system, and related personal information management system), and system management (security management, performance management, access user personal information management, fault management, etc.).

The overall model of the digital resource platform for ideological and political classroom teaching constructed in this research is as follows (Figure 4).

The learning mode of the digital resource platform for ideological and political classroom teaching is shown in Figure 5.

The production and development of the digital resource platform for ideological and political classroom teaching mainly include six stages: analysis and topic selection, design and planning, character resource collection and sorting, processing and production, platform construction, and evaluation and modification, as shown in Figure 6.

Audio, video, and video materials are the correct way to display the correct technical actions with background sounds and the combination of audio and video. The video part of the resource platform comes from the TV collection and self-recorded technical and tactical video pictures, which are self-shooting videos and from the internet. Among the channel guidance, audio and video digital resources use three storage formats, namely, AVI format, MPEG format, and streaming media format. The AVI format is used in the computer system, the MPEG format is used to separately enjoy larger video materials, and the streaming media format is used for real-time transmission and provision of video materials for real-time teaching on the internet and WeChat platform.

The animation materials of the resource platform are based on the characteristics of ideological and political teaching, and the video materials are analyzed and compared [22, 23]. The use of animation materials can more intuitively show the changes in ideological and political teaching in a two-dimensional space. The formats used for animation materials are GIF format, flash format, AVI animation format, and FLI/FLC animation format. The development of ideological and political classroom teaching resource construction network platform and WeChat platform mainly provide a complete set of network support for ideological and political teaching. Users upload instructional videos through the network platform. When the videos of instruction have been properly uploaded, any user will be able to view them, learn from them, and comment on them through the network. Students' time is saved because the construction of online teaching resources organizes technologies, theories, and cutting-edge consultations in detail. This not only achieves the purpose of allowing students to learn whenever and wherever they want, but it also makes it easier for students to quickly learn new skills and master new knowledge. Teaching information may be more quickly and easily sent through the network platform and the WeChat platform, and students can receive personalized instruction and guidance through one-on-one interactions with their teachers, as shown in Figure 7.

The framework structure of the WeChat public platform of the digital resource platform for ideological and political classroom teaching is shown in Figure 8.

The text material is as follows: it is mainly composed of textual materials summarized, edited, written, sorted, and collected from the collected research results related to ideological and political movements. Picture material is as follows: it mainly comes from self-photographed, internet, and ideological and political-related magazine pictures, and relatively accurate and high-resolution pictures of competitions and exercises. Moreover, according to the needs of the page, the pictures are processed and organized in a unified manner by using tools. Video material is as follows: it is a way of intuitive display of reasonable technical means. The video part of the WeChat platform of ideological and political classroom teaching digital resources comes from the collection of the internet and self-recorded technical and tactical video pictures.

The client is unique to each user, is used to conduct front-end functions, and because of its high reaction speed, it can fully utilize the client PC's processing resources. The client can handle a large amount of work before submitting it to the server. This system's student terminal primarily performs the following functions. (1) The student terminal validates fingerprint data. To begin, the teacher must launch the teaching assistant system service, and students must check attendance using the USB-connected fingerprint collector, log in to the student terminal, and enter the student ID, password, and fingerprint attendance information to gain access to the teaching assistant system. Following successful authentication, the interface will reveal student information such as student ID, name, test time, and other details. When the teacher prepares for the test, he or she sets up the corresponding test paper, on which the pupils can answer the questions. The setting status is waiting for the test when it has been performed. When the status is set to “start of test,” students can begin answering questions. (2) Students' classroom tests. To control the start of the examination, the teacher configures the test room, students, and test paper information on the server. After completing the related subjective and objective questions, students can submit their responses when the examination begins. If students come across unclear questions, they can mark them first and then return to respond once they have completed the confirmed questions.

The login module is mainly responsible for the functions of student login identity verification and authorization confirmation. Students taking the examination must log in on the student side. Before logging in, first, the teacher needs to make relevant configurations in the teacher's backend, that is, to provide the students with the login permission for the examination. Second, students must first enter their fingerprint information into the teacher's computer through the fingerprint collector to save it. The login process is shown in Figure 9.

## 5. Performance Analysis of Ideological and Political Classroom Teaching System Based on Digital Sensor Technology

This study constructs an ideological and political digital teaching system based on digital sensor technology, and uses digital sensor technology to improve the traditional teaching model to improve the quality of ideological and political classroom teaching. On this basis, this study conducts a performance test on the system, which mainly analyzes the digital effect and the improvement of the quality of ideological and political education. First, this study evaluates the digital effect of ideological and political classrooms, and obtains the results shown in Table 1 and Figure 10.

From the above experimental research, we can see that the ideological and political digital teaching system constructed in this study can reliably transform the ideological and political classroom teaching into a digital mode. Afterward, the ideological and political teaching system based on digital sensor technology is evaluated for teaching effect, and the results obtained are shown in Table 2 and Figure 11 below.

From the above experimental research, we can see that the ideological and political classroom teaching system based on digital sensor technology constructed in this study has certain value.

## 6. Conclusions

It is now a problem that needs to be studied and resolved as quickly as possible. This problem is how to reform the teaching of ideological and political theory courses that are offered in colleges and universities so that they can occupy the position of network ideological and political education and improve the pertinence and effectiveness of ideological and political teaching. Based on the findings of the inquiry and analysis of the existing situation, it appears that the current response of college students as a whole to “ideological and political courses” is not the optimal answer. The ideological and political education that is currently being provided in the higher education institutions of our nation is essentially the implementation of a “unilateral policy.” This means that the primary method of instruction is indoctrination and narration, which is devoid of interest, diversity, and abstraction. Some college students with higher educations have clear ideological, political, ethical, and value contradictions as a result of the “indoctrination” of boring and empty theories. This is often the result of the “indoctrination” of boring and useless theories. In addition, the “main ideas” that these kids adhere to are unmistakable, yet the daily actions that they exhibit are exasperating.

## Figures and Tables

**Figure 1:** Schematic diagram of spectrum leakage.

**Figure 2:** Schematic diagram of the fence effect.

**Figure 3:** Technical roadmap for the construction of a digital resource platform for ideological and political education.

**Figure 4:** The overall model diagram of the digital resource platform for ideological and political classroom teaching.

**Figure 5:** The learning mode of the digital resource platform for ideological and political classroom teaching.

**Figure 6:** The development stage of the digital resource platform for ideological and political classroom teaching.

**Figure 7:** The design stage of the WeChat platform of digital resources for ideological and political classroom teaching.

**Figure 8:** The framework structure of the WeChat public platform of the digital resource platform for ideological and political classroom teaching.

**Figure 9:** Login flowchart.

**Figure 10:** Statistical diagram of evaluation of digital effect of ideological and political classroom.

**Figure 11:** Statistical diagram of the evaluation of the teaching effect of the ideological and political classroom system based on digital sensor technology.

**Table 1:** Statistical table of evaluation of digital effect of ideological and political classroom.

Number	Digitizing	Number	Digitizing	Number	Digitizing
1	95.3	28	91.6	55	95.0
2	93.2	29	88.3	56	95.2
3	93.9	30	96.1	57	88.7
4	87.7	31	94.0	58	83.2
5	88.5	32	93.9	59	91.9
6	88.2	33	92.7	60	90.6
7	94.4	34	88.9	61	85.7
8	89.9	35	86.3	62	87.0
9	96.3	36	88.1	63	82.8
10	96.6	37	89.6	64	86.2
11	88.0	38	89.8	65	85.4
12	93.8	39	84.2	66	96.8
13	88.6	40	91.5	67	87.4
14	89.5	41	92.7	68	91.9
15	93.4	42	82.3	69	83.7
16	92.8	43	86.1	70	93.2
17	83.3	44	96.4	71	86.9
18	86.5	45	86.7	72	90.7
19	83.1	46	88.5	73	96.9
20	82.2	47	83.2	74	95.9
21	94.5	48	85.7	75	96.4
22	94.8	49	94.1	76	88.7
23	93.0	50	85.0	77	90.9
24	91.9	51	96.5	78	84.2
25	92.1	52	89.4	79	90.9
26	91.2	53	88.3	80	91.4
27	86.2	54	86.4	81	90.2

**Table 2:** Statistical table of the evaluation of the teaching effect of the ideological and political classroom system based on digital sensor technology.

Number	Teaching effect	Number	Teaching effect	Number	Teaching effect
1	89.2	28	91.6	55	88.1
2	93.0	29	90.0	56	88.6
3	91.7	30	92.4	57	93.3
4	90.2	31	90.6	58	92.6
5	92.6	32	92.1	59	90.0
6	88.8	33	93.9	60	91.1
7	89.5	34	91.2	61	93.3
8	89.2	35	92.5	62	92.4
9	90.5	36	92.6	63	88.0
10	93.6	37	88.6	64	93.3
11	92.3	38	90.9	65	88.2
12	90.9	39	89.1	66	92.5
13	89.7	40	93.1	67	92.8
14	92.4	41	92.5	68	88.8
15	88.5	42	90.2	69	91.5
16	91.8	43	93.5	70	90.9
17	89.2	44	91.3	71	89.8
18	89.9	45	91.9	72	89.2
19	92.1	46	91.5	73	93.8
20	92.2	47	93.6	74	91.8
21	88.4	48	89.8	75	93.1
22	92.5	49	88.1	76	92.4
23	89.5	50	92.7	77	90.1
24	93.0	51	91.8	78	90.3
25	93.2	52	92.2	79	88.9
26	91.0	53	94.0	80	88.2
27	89.8	54	89.1	81	93.0

## Data Availability

The data used to support the findings of this study are included within the article.
